This article has been retracted.

# An Artificial Intelligence-Based Bio-Medical Stroke Prediction and Analytical System Using a Machine Learning Approach

**DOI:** 10.1155/2022/5489084

**Published:** 2022-10-12

**Authors:** R. Pitchai, Bhasker Dappuri, P. V. Pramila, M. Vidhyalakshmi, S. Shanthi, Wadi B. Alonazi, Khalid M. A. Almutairi, R. S. Sundaram, Ibsa Beyene

**Affiliations:** ^1^Department of Computer Science and Engineering, B V Raju Institute of Technology, Narsapur 502313, Telangana, India; ^2^Department of Electronics and Communication Engineering, CMR Engineering College, Kandlakoya 501401, Telangana, India; ^3^Department of Computer Science Engineering, Saveetha School of Engineering, Saveetha Institute of Medical and Technical Sciences, Chennai 600124, Tamil Nadu, India; ^4^Department of Electronics and Communication Engineering, SRM Institute of Science and Technology, Ramapuram, Chennai 600089, Tamilnadu, India; ^5^Department of Computer Science and Engineering, Kongu Engineering College, Perundurai 638060, Tamil Nadu, India; ^6^Health Administration Department, College of Business Administration, King Saud University, P. O Box: 71115, Riyadh 11587, Saudi Arabia; ^7^Department of Community Health Sciences, College of Applied Medical Sciences, King Saud University, P. O. Box 10219, Riyadh 11433, Saudi Arabia; ^8^Department of Health Sciences, University of Texas, TX, USA; ^9^Department of IT, Mettu University, Mettu, Ethiopia

## Abstract

Stroke-related disabilities can have a major negative effect on the economic well-being of the person. When left untreated, a stroke can be fatal. According to the findings of this study, people who have had strokes generally have abnormal biosignals. Patients will be able to obtain prompt therapy in this manner if they are carefully monitored; their biosignals will be precisely assessed and real-time analysis will be performed. On the contrary, most stroke diagnosis and prediction systems rely on image analysis technologies such as CT or MRI, which are not only expensive but also hard to use. In this study, we develop a machine learning algorithm for the prediction of stroke in the brain, and this prediction is carried out from the real-time samples of electromyography (EMG) data. The study uses synthetic samples for training the support vector machine (SVM) classifier and then the testing is conducted in real-time samples. To improve the accuracy of prediction, the samples are generated using the data augmentation principle, which supports training with vast data. The simulation is conducted to test the efficacy of the model, and the results show that the proposed classifier achieves a higher rate of classification accuracy than the existing methods. Furthermore, it is seen that the rate of precision, recall, and *f*-measure is higher in the proposed SVM than in other methods.

## 1. Introduction and Related Works

The 4^th^ Industrial Revolution has arrived, bringing with it a wide range of businesses and research fields and huge opportunities as well as substantial challenges. These might be thought of as two sides of the same coin. Because of the role they play in the Fourth Industrial Revolution, artificial intelligence, big data, the Internet of things (IoT), and cloud computing have become popular topics of discussion in the healthcare business [1–4]. As a result of the Internet of things (IoT), medical devices and facilities now can send and receive biosignals, medical records, and even genetic data over the Internet. The rapid ageing of the world population will lead to an increase in the prevalence of chronic diseases as well as an increase in the cost of providing medical care [5]. As a means of preparation, national healthcare systems are shifting their emphasis away from the treatment of illness and disease and toward the promotion of overall health and well-being. The different types of health data that may be easily analysed to the creation are shown in Figure 1.

- Big data are personal health records (PHRs)
- Electronic medical records (EMRs)
- Genomic information

Classifier is the block that is used to classify the different dimensions of the image. This was very useful to identify the different stroke locations and depth of the stroke. Even though enormous volumes of medical data have been gathered and stored over the years, the data have not yet been utilised to its full potential. Combining the technologies of big data and artificial intelligence (AI) enables the development of novel intelligent medical solutions, as shown in Figure 2.

- Precision healthcare services
- Predictive health care services

They are both examples of those that are conceivable. However, it is currently difficult to derive relevant insights from multiple types of healthcare data by merging them. Because of recent developments in computer infrastructure and the appearance of multiple AI frameworks in information and communication technology (ICT), AI-based digital healthcare analysis has recently become more complex and feasible. A new method called smart healthcare allows for the remote management of people's health by utilising ICT and large amounts of medical data [6].

According to the World Health Organization, the leading causes of death worldwide in 2016 were malignant neoplasms (often known as cancer) and heart disease. In 2016, diseases related to strokes were responsible for 5.7 million fatalities, making them the third greatest cause of death overall. In the year 2016, most of the people were affected by the stroke, and this stroke played the critical factor to increase the death ratio [7]. This will result in the death of brain cells. It is more common for elderly people to suffer from strokes, which can result in a variety of symptoms, including hemiplegia, slurred speech, and loss of consciousness, in addition to various forms of brain damage. Because of them, adults are at risk of severe disability and possibly death. If an impending stroke can be recognised or predicted in its early stages, it may be feasible to significantly mitigate its effects [8–10]. Several risk factors for stroke have been established through the course of a great number of investigations and clinical trials. Tobacco use, high blood pressure, diabetes, and obesity are all preventable risk factors for stroke that can be managed and treated to lower the risk of having a stroke. Both medical and personal efforts, as well as immediate research and steps, are required to be performed at the national level to prepare for a forecasted increase in more stroke disorders as a result of the worldwide trend toward an older population [11]. People who think they are having a stroke should go to the hospital immediately, be examined by a stroke doctor, have an X-ray of the brain taken, and receive anticoagulation as soon as possible. They should not feel that they are too old for treatment. Treatment given within three hours of stroke is most effective; treatment given after 4.5 hours maximizes yield. Studies are testing this because it is unclear about the effectiveness of treatment given after that. Data from studies are needed to determine whether the benefit of anticoagulation therapy outweighs the risk of bleeding in patients with mild stroke.

It may be difficult to anticipate stroke symptoms or outbreaks using risk factors because the definitions of various risk variables and methods for correlating the likelihood of various diseases occurring are variable. When it comes to determining the prognosis of an illness such as stroke, placing all of your faith in the risk factors alone presents several challenges. The Framingham Heart Study proposed a methodology for predicting the risk of stroke based on a prospective cohort study of cardiovascular illness [12, 13]. Especially, if this treatment is given within three hours of stroke onset, older people are benefited as much as younger people. Adding aspirin to anticoagulants increases the risk of bleeding; so, it should be avoided. Further analysis of individual data factors, such as pretreatment CT scans of patients' brains and different treatment options rather than aggregate data, will reveal more.

It is difficult to recognise a stroke and the accompanying brain damage early on due to the wide variety of symptoms and categories that are associated with a stroke. It is a risk factor, the severity of which depends on the outcomes of prior medical exams. It is difficult to apply this to the multiple symptoms and prognoses of an elderly person (patient) before the beginning of a stroke because they show the predicted possibility of disease developing in the far distant future, which is approximately five to ten years away. People who are forced to work long hours can avoid problems if they exercise and eat healthy food in between their working hours. The researchers came to this conclusion by analysing the data of age and smoking and working hours of more than 143,000 people. That is, 1,224 people who worked more than 10 hours for more than 10 years had suffered a stroke. A well-planned diet, regular exercise, quitting smoking, and eating the right amount of food can make a huge difference in people's health.

Artificial neural networks, also known as ANNs, have been utilised in several studies for the diagnosis or prediction of strokes. Singh et al. [14] concluded that the ANN is capable of identifying people who are at risk of having a stroke. In that particular study, the backpropagation method was utilised to improve the accuracy of both prediction and diagnosis. Because of an artificial neural network, it was feasible to predict the risk of having a stroke using only 300 pieces of experimental data (ANN). The inquiry led to the creation of a model that is accurate 95.33% of the time for patients suffering from a stroke. In this particular instance, however, the primary focus is placed entirely on the precision of the forecast, which makes it challenging to analyse the underlying operational concept in finer detail. The researchers [15] looked at how well CT scans and clinical factors could predict the risk of cerebral haemorrhage occurring during the freezing treatment for ischemic stroke patients. By analysing CT images of 116 patients suffering from ischemic stroke, SVMs were successful in identifying nine out of sixteen patients with symptomatic cerebral bleeding.

They [16] employed the kernel function of SVM to update the parameter values of a prediction model for stroke risk. The variables that contribute to the risk of stroke were analysed. By making use of the RBF kernel function, this model was able to accomplish a degree of accuracy that was satisfactory. In contrast to early detection or the prediction of preoccurrence symptoms, the research that was conducted using SVMs focused on predicting severity and prognosis after an epidemic had already taken place. This system has several flaws, one of which is that its working principles are a mystery. This is because all it does is improve the precision of traditional stroke predictions. Because it relies on the findings of individual clinical diagnostic tests and CT scans, this method is unable to detect and forecast the presymptoms of stroke disorders based on real-time biosignals or life logs. In addition, it is not possible to determine whether or not a stroke disorder will occur. As a consequence of this, additional research, as well as clinical trials, are required to recognise strokes in their earliest stages. To address the limitations, Yu et al. [17] conducted an investigation and released research that made use of data mining techniques. According to research, a decision tree algorithm-based data mining classification approach was applied to automatically classify and interpret the results of the NIHSS in terms of the severity of the condition being measured. In addition, a fresh approach to the semantic interpretation of stroke severity was produced by carefully analysing the rules on the principle of motion. These rules offer further data for the C4.5 decision tree, and their analysis led to the development of a fresh approach. Because of the decision tree approach, the predictive model algorithm can only provide a limited interpretation of the data. As a result of this limitation, the predictive model is considered. Another study to predict the risk of stroke was conducted in [18], which looked at more than 50 potential risk variables. In this study, accurate stroke prediction was achieved with the application of data mining techniques such as the K-nearest neighbours algorithm and the C4.5 deception tree. The approach, like others that were used in prior studies, is not appropriate for the use in everyday life to detect and forecast presymptoms of stroke. The processing and interpretation of time-series data is a common application of recurrent neural networks, also known as RNNs, in the field of deep learning. RNNs use circulatory neural networks as a component of the current learning process. These networks are founded on the results of prior phases of the learning process. Because the outputs of recurrent neural network structures, also known as RNNs, include information about the outcomes of calculations that have been performed in the past, RNNs can acquire knowledge of sequential data.

Models such as Long Short-Term Memory (LSTM), which is also a class of the RNN, can manage the challenge of computing and reducing values when wrong values are sent to the neural network layer. This allows these models to overcome the structural defects that are present in the current RNN. This LSTM was initially proposed in [19] in the year 1997. Within these neural networks, the sigmoid and tan(*h*) layers, in conjunction with the cell states, input gates, forget gates, and output gates, are responsible for generating vector output values at each of these gates. The cells of the LSTM are responsible for learning how to recognise and protect essential inputs often known as input gates. The cells that make up the LSTM learn how to remove them whenever it becomes necessary to do so. An EHR risk factor analysis has been used recently to predict LSTM-based cerebrovascular diseases. This represents a new study trend in the field of LSTM research. In particular, Chantamit-o-pas and Goyal [20] discovered that the LSTM algorithm is the best at predicting any cerebrovascular disease or stroke by using ICD-10 codes and other pertinent risk factor patterns from EHRs. A method for predicting the transition from an ischemic stroke to a hemorrhagic one was proposed in [21] using the LSTM model (HDM). It was determined that diffusion and perfusion-weighted magnetic response photographs were necessary to create the LSTM network topology. A comparative analysis of 155 patients with acute stroke who participated in clinical trials revealed an accuracy rate of 89.4%. Even though these studies have shown that the LSTM can predict strokes, they have still relied on data such as EHR. Because no study of this kind has been conducted in this field, it is not possible to forecast or evaluate the likelihood of a stroke by analysing real-time biosignals generated by everyday activities such as walking or driving. A unique strategy that is based on real-time biosignals is required as an alternative to the existing traditional methods that are currently being used to predict strokes. Because of an artificial neural network, it was feasible to predict the risk of having a stroke using only 300 pieces of experimental data (ANN). The inquiry led to the creation of a model that is accurate 95.33% of the time for patients suffering from a stroke. In this particular instance, however, the primary focus is placed entirely on the precision of the forecast, which makes it challenging to analyse the underlying operational concept in finer detail. The goal of this research is to build a machine learning system capable of predicting brain strokes. This forecast is based on information derived from real-time EMG data. The support vector machine (SVM) classifier is trained with simulated data first and then evaluated with real-world data.

## 2. The Proposed Method

In this study, we develop a machine learning algorithm for the prediction of stroke in the brain and this prediction is carried out from the real-time samples of electromyography (EMG) data as illustrated in Figure 3. The study uses synthetic samples for training the support vector machine (SVM) classifier, and then, the testing is conducted in real-time samples. To improve the accuracy of prediction, the samples are generated using the data augmentation principle, which supports training with vast data.

Most strokes are caused by a blood clot in an artery in the brain. Timely treatment with thrombolytic drugs can help restore blood flow before a large stroke occurs and improve recovery after a stroke. However, death can occur from severe bleeding in the brain caused by anticoagulants.

### 2.1. SVM Classifier

Binary linear classifiers are examples of supervised linear classifiers. These classifiers are often known as support vector machines (SVMs). Support vector machines can be modified to conduct nonlinear classification, and with the addition of a few extra techniques, they can perform classification on an endless number of different classes. By utilising a support vector machine, it is possible to generate an arbitrary hyperplane between two different sets of vectors that can be differentiated linearly. In particular, the hyperplane that minimizes the distance between itself and any point in either of the clusters is the one we are interested in. When classifying a testing point, the side of the calculated hyperplane, on which the point lies, is taken into consideration. It is possible to train support vector machines to function in other contexts in addition to the two linearly distinct classes for which this straightforward approach is effective.

### 2.2. Nonlinearly Separable Classes

If the two classes cannot be linearly separated using this approach (no hyperplane can be generated that perfectly splits the classes on either side), then you will not be able to use this method. In this scenario, you will need to construct a soft margin that will almost exactly split the data into two distinct classes. During this step of the process, cost functions are determined. The most significant component of this cost function is referred to as the hinge loss function. If a point is located on the appropriate side of the hyperplane, then the value of this function is equal to zero. However, if the point is located on the incorrect side of the hyperplane, then the value of this function is proportional to the distance from the hyperplane. It is the hinge loss function that is averaged over all of the data points, plus a parameter that defines the trade-off between increasing the number of points that are on the correct side of the hyperplane and maximizing the smallest distance that correct points are from the hyperplane. By lowering this cost function, it is possible to generate a classification hyperplane with respectable results. This method performs relatively similar to the classic SVM algorithm in situations when the input can be linearly separated, and it continues to function admirably in situations where the input cannot be linearly separated.

There are two primary methods for classifying a large number of classes when using support vector machines; both of these methods function by establishing several binary classification support vector machines and obtaining a consensus vote among them to perform classification, respectively. Both of these methods use support vector machines. It is possible to train a support vector machine, often known as an SVM, for each class. When utilising this SVM, the selected class is considered to be one class, while the other data points are considered to be the other class. To put it another way, each sub-SVM is responsible for determining whether or not a particular point belongs to the class in question or another class. The class to which the point is assigned is determined by the category that the person making the assignment feels most strongly about. In the alternative approach, a classifier is designated for each possible combination of classes. When classifying points, we look at which of two possible classes is supported by the greatest number of pair wise classifiers.

### 2.3. Performing Nonlinear Classification

It is possible, with the help of a hyperplane, to split up some data sets into two categories that do not naturally correspond to one another. In this scenario, it does not matter which SVM algorithm is utilised; the result will be the same: an inaccurate classification of the data. In this section, the data can be altered to appear in a higher-dimensional feature space, which enables the classes to be differentiated from one another straightforwardly. You are engaging in the kernel trick at this very moment. When mapping points in two dimensions, you can make use of a Gaussian function, which positions points closer to the centre of the data higher on the map than points further away from the centre.

### 2.4. Data Augmentation

The capacity of data augmentation to improve photographs may be traced back to its earliest applications, such as horizontal flipping, colour space augmentation, and random cropping. Using these adjustments, which encode many of the invariances discussed earlier, is one way to relieve some of the challenges associated with image recognition. In this review, several different types of learning techniques, including geometric, colour space, kernel, mixing, random erasing, feature-space, adversarial training, GAN-based (GAN represents the Gathering and Additive Node. This node is an interconnection node between the two end points of different clusters. This node was helpful here to gather the various attributes and transmit the details between the end points), neural style transfer, and meta-learning, were identified as areas for improvement. In this section, we will explain how each method of enhancement functions, report the findings of our trials, and discuss some of the restrictions imposed by the enhancements.

### 2.5. Geometric Transformations

This section goes over a lot of different image processing functions, including geometric transformations, among other things. One method to categorise these enhancements is based on how straightforward it is to put them into action. A comprehensive understanding of these changes is required to lay a solid foundation for additional research into the various ways of data augmentation. Within the context of this conversation, we will also talk about the many different geometric augmentations in terms of their safety. When evaluating the safety of data augmentation methods, one must consider the likelihood that the label will continue to exist in its original form after the change. It may be possible, with the use of a nonlabel preserving transformation, to improve the capability of the model to offer a response indicating that it does not have confidence in its prediction. On the contrary, this would require postaugmentation labelling that is more precise. If the image label is [0.5 0.5] after a modification that does not preserve the label, the model may be able to generate predictions with a higher level of strong confidence. On the contrary, the process of constructing enhanced labels for every nonsafe data augmentation is both time-consuming and expensive.

Because it is difficult to produce revised labels for data that has been updated, augmentation needs to be regarded as safe before it can be implemented. Because augmentation policies need to be tailored to each industry, it might be challenging to generalise them. In the process of image processing, there is not a single function that does not, at some point in time, result in a transformation that modifies the labels. This demonstrates how challenging it can be to build generalizable augmentation rules due to the data-specific nature of their construction. This consideration is necessary because of the geometric augmentations that are detailed later.

### 2.6. Flipping

The horizontal axis is the one that is typically flipped, as opposed to the vertical axis, which is the more uncommon choice. Including this augmentation in datasets such as CIFAR-10 and ImageNet is one of the easiest and most effective ways to improve their accuracy. This is not a label-preserving transformation and therefore should not be used on datasets involving text recognition such as MNIST or SVHN.

### 2.7. Colour Space

Tensors are the common format for the recording of the dimensions of digital image data, which include height, breadth, and colour channels. Increasing the vibrancy of individual colour channels is another strategy that can be easily put into action. A straightforward method for improving a picture colour can be accomplished by isolating a single colour channel, such as R, G, or B. Quickly converting an image into its representation in a particular colour channel can be accomplished by isolating the matrix of one colour channel and adding the zero matrices from the other channels. Performing matrix operations on the image RGB values is all that is required to either increase or decrease the brightness of an image. Histograms of colours are employed in the process of developing increasingly intricate colour augmentations. Changing the intensity values of these histograms is the method that is used by photo editing software to make adjustments to the lighting.

### 2.8. Cropping

When processing picture data that has mixed height and width dimensions, cropping an image centre patch might be a valuable step to take as part of the processing workflow. A translation can also be imitated by employing random cropping, which generates an effect that is analogous to that of a translation. However, random cropping will result in a reduction in the image dimensions, for example, from (120,120) to (256,256). Translations will keep the image's spatial dimensions intact (224,224). Depending on the cropping threshold that was used, this modification may or may not preserve the labels of the original data.

### 2.9. Rotation

To execute rotation augmentations, the image is either rotated to the right or left along an axis that ranges from 1 degree to 359 degrees. Here, the term degree represents the image dimensional places. This was very helpful here to identify the stressful locations of the patients. As a consequence of this, the security provided by rotational enhancements is heavily reliant on the rotation degree parameter. Applications such as MNIST that need digit recognition do not keep the original data label after it has been transformed if the rotation degree is increased.

### 2.10. Translation

To eliminate any positional bias in the data, images can be rotated to the left or right, moved up or down, or shifted in any of these four directions. If all of the images in a collection are centred, for instance, a face-recognition model would have to be validated using photographs that are centred to the same degree. Depending on the direction in which the original image is translated, it is possible to fill the space that is left behind with either a set value, such as 0s or 255s or with random or Gaussian noise. One of these alternatives is superior to the other. The spatial dimensions of the postaugmentation image can be preserved with the help of padding.

### 2.11. Noise Injection

In most cases, a Gaussian distribution of arbitrary values is used in the noise injection process. The training of CNNs to learn more detailed characteristics can be helped by increasing the amount of noise that is present in the images. Using geometric modifications to reduce biases in training data is a wonderful way to go about it. The distribution of the training data could be very different from the distribution of the testing data in a variety of ways. If there are any placement biases in the dataset, such as in a facial recognition dataset when all of the faces are exactly centred, this is a good technique to use. Geometric transformations are helpful not only because of their ability to counteract the effects of positional biases but also because of how straightforward it is to put them into practice.

Because there are so many libraries to choose from, beginning image editing techniques such as horizontal flipping and rotation can be accomplished with relative ease. As a consequence of the alteration of the geometry, additional resources, including memory, additional time for training, and additional costs associated with calculation, are required. To verify that the image label has not been changed in any way, it is necessary to manually analyse any geometric changes that have been made, such as translation or arbitrary cropping. Last but not least, in many of the application disciplines that have been addressed, such as medical image analysis, biases are more complicated than positional and translational changes. These biases are that which differentiate training data from testing data. As a direct consequence of this, the application window for geometric transformations is quite limited.

### 2.12. Colour Space Transformations

The image data are encoded using three stacked matrices, each of which has a height and width that is proportional to the height. Each RGB colour value is represented by its separate dot in these matrices. When it comes to picture identification, one of the most common types of roadblocks is bias in the illumination. It is simple to understand why colour space alterations, sometimes referred to as photometric transformations, are effective. Looping through the images in question is all that is required to swiftly adjust the pixel values of photographs that are either too bright or too dark. A more straightforward method for manipulating the colour space is to splice off the various RGB colour matrices. In a transformation, pixel values can also be constrained to fit within a range with a minimum value and a maximum value, respectively. The inherent colour representation of digital photos makes a wide variety of improvements possible to be made to the quality of the images.

Alterations to the colour space can also be generated through the use of image editing software. A colour histogram is a graphical representation of how the pixel values of an image are distributed across each of the RGB colour channels. Increasing the vibrancy of individual colour channels is another strategy that can be easily put into action. One method to categorise these enhancements is based on how straightforward it is to put them into action. By adjusting the values of this histogram, it is possible to apply various filters to an image. This study, which was conducted using only data, revealed that self-employed people, chief secretaries, managers, etc., do not suffer from stroke even if they work long hours, while those who work long hours at irregular hours and at night are severely affected.

## 3. Results and Discussion

In this section, the process of monitoring and collecting biosignal data to verify the proposed AI-based stroke sickness prediction system is broken down in detail. The data from a real-time electromyogram will be the primary biosignal that is utilised. An electromyogram, or EMG, is a diagnostic tool that can be used to determine the speed of nerve conduction or record electrical activity within the muscle itself. An EMG does this by using electrodes to apply electrical stimulation to a muscle or nerve. According to the findings of several studies that utilised EMG, there is a little imbalance in the body both before and after a stroke, as well as imbalances in gait and locomotion. In this study, we investigate biosignal abnormalities as well as gait issues, both of which have been linked to an increased risk of stroke. Our stroke rehabilitation group consisted of patients aged 70 and older who had received a stroke diagnosis during the previous 30 days. Three hundred patients in the rehabilitation division fulfilled our requirements. Signals such as electrocardiography, electromyography, speech recordings, electroencephalography, and foot pressure were among the many that were collected for processing.

Before any biosignal data was acquired, the sensors were put through a series of rigorous tests to guarantee that they were in proper working order. Data were collected from a total of 300 patients, none of whom had survived a stroke and all of whom were considered to be in the normal group. Each patient was put through a variety of exercises that included standing, walking, sitting, raising their arms, and even sleeping to simulate actions that people do regularly. Before beginning the actual measuring technique in each situation, one practise run was provided for each individual to ensure accurate results. The first values that were collected and gathered could have been influenced by human noise caused by a subject's tension or discomfort; as a result, these values were not included as experimental data. Exerting senior citizens over and over again in trials is a waste of their time, which is why the most recent measurement methods were left out. Through the use of the Bluetooth protocol, each piece of biosignal data was transmitted instantly and directly to the main server. The data from the gateway bio-signals is sent to the server that accumulates and predicts bio-signals via the Wi-Fi connection protocol. A medical doctor oversaw the entirety of the measurement experiment and a fresh set of measurements was taken to check if any of the collected biosignal data was corrupted or destroyed. A bogus value consisting of four bytes of sampling rate in voltage was utilised for the EMG data that were transmitted from each of the four EMG sites.

To detect neuromuscular abnormalities and problems with balance, electrical activity in the muscles, as measured by EMG biosignals, is used. This activity can also be considered a muscle reflex. In this particular work, EMG biosignals are utilised to construct a machine learning model for stroke prediction. The characteristics are arrived at by deriving them from the raw muscle data of the biceps and gastronomies muscles. Variables obtained from EMG raw data were incorporated into tests of prediction models based on machine learning as well as multidimensional analyses. When extracting characteristics, data points were obtained by dividing the raw data into 0.1-second units. Since the variability of muscle movement was deemed acceptable at 1500 Hz per second EMG, this division was used. The procedures described in this research were utilised in the collection of the data. In our investigation, we relied entirely on the electromyographic (EMG) biosignals that were captured at the time of our scenario, which encompassed activities such as standing, walking, stretching one arm, and even sleeping. Only the data regarding walking was analysed, even though there existed a wide variety of experimental data. In Tables 1 and 2, it shows the classification accuracy used on the training and testing set.

This section is focused on the findings related to the classification of elderly stroke patients and nonstroke patients using the LSTM, which is based on a recent neural network (RNN). The development and evaluation of prediction models were based on the data collected from 271 stroke patients and 271 healthy individuals, respectively. After being randomly separated from the data sets used for learning, the data that were not put to use for learning were transformed into test sets. The experiment and the analysis had a ratio of 70/30 and 80/20, respectively. These ratios were used to divide the experiment and the analysis.

In Figures 4to 7, the result achieved using the proposed method with several metrics has been discussed. By collecting EMG bio-signals while the subject was walking, the prediction accuracy of stroke disorders of 90.38% was reached using the machine learning algorithm and random forest, and 98.958% was acquired using the deep learning LSTM method. In the course of this inquiry, EMG healthcare devices were utilised to gather real-time data at a frequency of 1500 Hz from a total of four different sites, including the left and right biceps fenestrum as well as the gastrocnemius muscle. Because it enables medical professionals and hospitals to take preventative measures for the early detection and diagnosis of stroke diseases in patients who are in the danger group, using these real-time biosignals to analyse and forecast stroke illnesses is a wise strategy. The model that was developed by machine learning and deep learning should be thoroughly analysed by medical staff, electronic medical records, clinical data, emergency blood test and MRI information, and other relevant data to ensure accurate stroke illness analysis and forecasts. This will allow for better patient care. As a consequence of this, rather than placing all of their faith in the AI-based model that was built as a result of this body of work, researchers ought to incorporate studies that make use of medical expertise and clinical experimental data to forecast stroke disease.

Because of the experiments done in this study with EMG biosignals just while walking, the prediction of multimodal biosignals such as EEG and ECG should also be taken into consideration. The ultimate goal was to ensure that intensive research into the early diagnosis and prognosis of strokes and other chronic diseases, such as diabetes and heart disease, would be carried out using signaling as the primary method. Using the experimental findings from this study that are based on EMG, medical practitioners can effectively foresee and identify stroke illnesses. Furthermore, the preliminary findings suggest that AI approaches can be utilised to assist in the diagnosis of diseases purely in everyday life.

## 4. Conclusion

The purpose of this study is to construct a machine learning system capable of predicting strokes in the brain using real-time EMG data. Then, the SVM classifier is trained using simulated data and is then tested using actual data. The samples are generated by the application of the notion of data augmentation, which makes it easier to train with a substantial quantity of data. When the simulation is run to check if the model performs as anticipated, the results show that the proposed classifier is more accurate than the approaches that are currently being used. In the cutoff point, the proposed model achieved 91.77% of accuracy, 90.28% of precision, 91.44% of recall, and 91.12% of *F*1-Score. The proposed model was getting a high level while compared with other models. Furthermore, the SVM accuracy, recall, and *f*-measure are all higher than those of the competing approaches.

## Figures and Tables

**Figure 1:** Different types of health data.

**Figure 2:** Novel intelligent medical solutions.

**Figure 3:** The Proposed classification model.

**Figure 4:** Accuracy.

**Figure 5:** Precision.

**Figure 6:** Recall.

**Figure 7:** F-measure.

**Table 1:** Classification accuracy on the training.

Signal of patient	TP	TN	FP	FN
20	592	5	4	1
40	1394	21	3	10
60	795	26	6	3
80	204	14	9	10
100	687	23	12	8
120	450	21	3	9
140	609	1	3	1
160	434	29	8	7
180	936	18	6	12
200	2415	18	19	3
220	561	15	2	15
240	558	24	12	4
260	1236	10	11	8
280	367	11	7	1
300	611	15	4	2

**Table 2:** Classification accuracy on testing.

Signal of patient	TP	TN	FP	FN
20	593	2	5	2
40	1383	28	11	6
60	802	21	6	1
80	216	12	6	3
100	686	23	9	12
120	438	23	12	10
140	595	14	2	3
160	442	19	16	1
180	937	18	9	8
200	2429	10	6	10
220	561	19	9	4
240	563	18	12	5
260	1233	12	15	5
280	349	18	11	8
300	593	10	20	9

## Data Availability

The data used to support the findings of this study are included within the article and can be obtained from the corresponding author upon request.
